# Sports Training Teaching Device Based on Big Data and Cloud Computing

**DOI:** 10.1155/2021/7339486

**Published:** 2021-09-24

**Authors:** Gexin Chao, Wu Gang

**Affiliations:** ^1^Langfang Normal College, Langfang, Hebei 065000, China; ^2^Langfang Health Vocational College, Langfang, Hebei 065000, China

## Abstract

With the advent of the era of big data (BD), people have higher requirements for information, knowledge, and technology. Taking the Internet as the carrier, the use of cloud computing technology for distance education has become a trend. Our country's physical training teaching has also begun to change from traditional mode to modern mode. In order to improve the overall quality of our country's national sports, this paper studies the teaching device of sports training based on BD and cloud computing. This article mainly uses the questionnaire survey method, the experimental analysis method, the data analysis method, and the data statistics method to have an in-depth understanding of the research theme and uses swimming as an example to design the sports training device. 52% of people think that water in the ears and itching during swimming are more serious problems. After further understanding, an experimental design was carried out. Experimental studies have shown that the combination of BD and cloud computing can effectively solve the problems existing in the traditional teaching model, so as to achieve the goal of efficient and rapid development.

## 1. Introduction

Sports power is an important part of the Chinese dream. Under the background of the era of BD, our country's physical education reform and development direction have also undergone tremendous changes, and traditional physical education teaching models have gradually been eliminated. Utilize the distributed storage, distributed computing, machine learning, high availability, high scalability, and platform consistency of the cloud platform to achieve high availability and scalability of the sports training teaching device platform; use BD analysis technology to achieve sports training intelligent analysis of effects, which is a high requirement for physical education [1, 2]. Big data refers to a data set that cannot be captured, managed, and processed by conventional software tools within a certain time range. It is a massive, high growth rate and diversified information asset that requires a new processing mode to have stronger decision-making power, insight and discovery power and process optimization ability.

There are many researches on teaching devices for sports training based on BD and cloud computing, and many people have studied training devices for different sports activities in a targeted manner. For example, some people have conducted research on the problem that the leveling of the bunkers in the long jump project requires a large amount of work. According to the current existing technology, the low-cost long jump bunker electric leveling device is applied to the physical education teaching, which involves the field of sports training automation. It is a long jump training system based on force plate and digital runway [3]. Someone also proposed a physical education training device with a base and a basketball hoop. The basketball stand includes a support rod and a backboard, and the backboard is provided with a basket, which is convenient to use and has the advantages of convenient practice and no restriction [4]. In addition, Xu Meidong proposed that the “Volleyball Comprehensive Training Device” is a multifunctional teaching and training equipment used in volleyball teaching and training, and it plays an important role in volleyball teaching and training. It utilizes the rebound effect of the adjustable baffle on the ball to realize the tandem of serve, pass, cushion, and smash techniques, speeding up students' mastery of volleyball skills. Use the device that imitates the “arm block” to speed up students' mastery and in-depth study of spiking techniques. The positioning ring device is used to strengthen the students' mastery of volleyball pad and pass techniques and improve the accuracy of students' passing and padding. In the absence of equipment and limited volleyball courts, the density of students' practice has been increased in the classroom, which can help students learn volleyball techniques and tactics [5]. Cloud computing is a kind of distributed computing, which means that the huge data computing processing program is decomposed into countless small programs through the network “cloud” and then processed and analyzed through the system composed of multiple servers. These small programs get the results and return them to users. In the early days of cloud computing, in short, it was simple distributed computing, which solved the task distribution and merged the calculation results. Therefore, cloud computing is also called grid computing. Through this technology, tens of thousands of data can be processed in a very short time (a few seconds), so as to achieve powerful network services.

This article first collects data on some conceptual features of BD and cloud computing. Secondly, it analyzes the current sports items, then elaborates on the development and system design of digital sports, researches sports training monitoring devices, and finally takes swimming as an example to design and study virtual swimming device. Cloud computing is not a new network technology, but a new network application concept. The core concept of cloud computing is to take the Internet as the center and provide fast and safe cloud computing services and data storage on the website, so that everyone using the Internet can use the huge computing resources and data center on the network.

## 2. Sports Training Teaching Device Based on Big Data and Cloud Computing

### 2.1. Sports

Countries all over the world are classified according to their own characteristics and habits. The Soviet Union and some Eastern European countries divided all sports and contents into games, gymnastics, sports (athletics), and travel. Japan is generally divided into games, athletics, performance sports, and forms of sports. For specific application, more detailed classification can be carried out according to different purpose requirements. Sports means are subordinate to the purpose and task of sports. The selection of sports means should start from specific tasks, vary from person to person, suit measures to local conditions, be scientific and reasonable, and focus on practical results. In order to strengthen the body and entertain the body and mind, sports have been valued since ancient times. There are many types of sports events. For details, please refer to Table 1.

As shown in Table 1, sports items are becoming more and more abundant, and people's competition in sports events is becoming more and more fierce. Common sports items include swimming, track and field, basketball, badminton, table tennis, and football. How to improve the ability of Chinese athletes and amateurs in sports items is the purpose and way for our country to participate in sports events and national physical and mental health for many years.

Sports are also classified, such as recreational sports, that is, recreational sports activities for the purpose of pleasurable body and mind. Generally, there are ball games, board games, and traditional national sports activities; mass sports, that is, sports to prevent diseases and strengthen physical fitness and sports activities for cultivating reserve talents; medical sports, that is, the use of sports methods to treat certain diseases and improve the physical activities of the body, generally including jogging, walking, and Tai Chi.

Sports is not only a social activity, but also a physical education activity. It can strengthen the body, provide social environment, and cultivate revolutionary friendship and sometimes is a life-saving magic weapon. For example, playing basketball not only requires physical fitness, but also requires people to have the spirit of teamwork and cultivate fighting friendship. Swimming not only is an international sporting event, but also can save lives in sudden falls. So this article also conducted a questionnaire survey on swimming enthusiasts.

### 2.2. Big Data

The value of big data is reflected in the following aspects: (1) Enterprises that provide products or services to a large number of consumers can use big data for precision marketing. (2) Small, medium-sized, and micro enterprises with a small and beautiful model can use big data for service transformation. (3) Traditional enterprises that must transform under the pressure of the Internet need to keep pace with the times and make full use of the value of big data.

#### 2.2.1. BD Concept and Characteristics

In recent years, big data has received extensive attention from the industry, academia, and even governments around the world. BD has had a significant impact on people's daily life, and it has received more and more attention from everyone. Whoever has the data has the initiative [6, 7]. There is no doubt that the arrival of BD not only brings huge scientific research and social, economic, and other values but also brings unprecedented opportunities to people. The definition of BD is also different. The definition of “BD” in Wikipedia mainly refers to a collection of data whose content cannot be captured, managed, and processed with conventional software tools within a certain period of time.

Although the precise definition of BD has not yet been unified, several characteristics of BD are generally recognized:

1. The amount of data (AOD) is huge. BD usually refers to the AOD that often reaches more than 1PB. The main reasons for generating such a large AOD are the wide use of various sensors and the types of data that can be collected; people are closely connected and need to communicate at low intervals throughout the period. In this way, the AOD exchanged grows exponentially.
2. There are many types of data. This is mainly due to the increase in the number and types of sensors, social networks, and smart devices and other wide-ranging applications. The types and composition of data are more complex. In addition to conventional relational data, there are also various types of web pages, audio, video, and documents. Formal, semistructured and unstructured raw data.
3. The flow rate is fast. Now is the information age. Data are updated and changed very quickly. Some information must be answered within a limited time; otherwise, it is out of date or invalid. The feature of BD emphasizes the rapid and dynamic changes of data and the formation of streaming changes.
4. The value density is low. A typical feature of BD is its low value density. The useful information hidden in the massive data does not increase with the exponential growth of the data volume. On the contrary, it is more difficult to obtain useful information. This requires the use of BD mining technology to process large data sets with low value density, so as to obtain useful data.
5. Accuracy of results: the results of BD processing must ensure certain credibility.

### 2.3. Cloud Computing

#### 2.3.1. Concept

Cloud computing (CC) is a widely used and mature technology, and its definitions are not the same. As per Wikipedia, CC integrates and encapsulates information technology resources into services and provides users with them. Users can obtain the services they need through network connections. CC is developed based on the integration of distributed computing, virtualization technology, network computing, and web services. Users can obtain resources on demand at any time without restriction and can handle large-scale data and problems [8]. CC adopts virtualization and multitenant technology. Virtualization is a resource processing technology that abstracts and transforms various physical resources such as servers, computers, and networks. It is a large-scale integration of resources. In terms of being a whole, it breaks the inseparable barriers between physical structures. Multitenant technology is a software architecture processing technology, which can ensure the independence and isolation of user data, and the premise for achieving this is that multiple users share the same system. These two technologies can be summed up in a nutshell as the sharing of physical resources by different users is the virtualization technology; the sharing of the same software or component resources by different users is the multitenant technology.

The resource data on the cloud system is very large, and the update speed of resource information is fast. If you want accurate and reliable dynamic information, you need effective ways to ensure the rapidity of information. The cloud system can effectively deploy dynamic information and also has the function of resource monitoring, which is conducive to the management of resource load and usage. Secondly, as the “blood” of resource management, resource monitoring plays a key role in the overall system performance. Once the system resource supervision is not in place and the information lacks reliability, other subsystems cite wrong information, which will inevitably have an adverse impact on the allocation of system resources. Therefore, it is urgent to implement resource monitoring. In the process of resource monitoring, as long as the agent is deployed on each cloud server, it can carry out configuration and supervision activities. For example, connect each cloud resource server through a monitoring server and then send the resource usage to the database in cycle. The monitoring server will analyze all resources and evaluate the availability of resources by integrating the effective information of the database, Maximize the effectiveness of resource information.

#### 2.3.2. Features

1. Huge scale: it is usually composed of tens of thousands or hundreds of thousands of services, and the scale is very huge.
2. Virtualization: users do not need to care about specific locations, they can obtain services through any location and various terminals, and resources are uniformly allocated by the system. For users, all requested resources come from the cloud, rather than a specific server.
3. High reliability: CC has multiple copies and computing nodes that can be easily interchanged. These technologies can ensure data redundancy and reliability. Good versatility: the same cloud can support different applications at the same time, rather than specific applications.
4. High scalability: Cloud is integrated from physical servers, computers, storage, and other equipment and realizes unified management. This model is very convenient for expansion and can easily meet the growth needs of user.
5. Low cost: the cost of a single cloud node is very low, and when integrated into the resource pool, the computing and storage capabilities are strong. For users, they only need to care about the services they want, instead of maintaining physical equipment, thereby saving a lot of maintenance costs. The resource pool is centralized and automated by professionals, which in turn can save a lot of costs and can support users to provide high-quality and low-cost services.

#### 2.3.3. Classification

According to the scope of deployment, CC can be divided into three categories: public cloud, private cloud, and hybrid cloud:

1. Private cloud: private cloud, also called exclusive cloud, is generally deployed inside an enterprise or organization, only provides services within the enterprise or organization, and is not open to the public. Private cloud has the characteristics of flexible configuration, easy maintenance, and management and at the same time has good privacy.
2. Public cloud: public cloud can provide services for organizations, enterprises, or individuals in need. It is generally provided by a dedicated cloud service provider. The cloud server provider deploys its own infrastructure, and users only need to request through their own terminal equipment. The service is sufficient, and the user generally has to pay a certain fee for the service.
3. Hybrid cloud: hybrid cloud is a mode that combines public cloud and private cloud. Using hybrid cloud can take advantage of the advantages of public cloud and private cloud. Services that require a high degree of confidentiality and high security are deployed on a private cloud; for general-purpose services, services that are not highly confidential and have insufficient resources can be deployed on a public cloud. The hybrid cloud deployment method can effectively shorten the construction period and save the construction cost and can not only meet the security requirements, but also meet the convenience requirements. Hybrid cloud provides many important functions that can benefit enterprises of all shapes and sizes. Its characteristics mainly include reducing cost, increasing storage and scalability, improving availability and access ability, improving agility and flexibility, and obtaining application integration advantages.

#### 2.3.4. CC Architecture

CC can link various resources to form a resource pool for users, realize resource sharing, and can easily expand. CC consists of three layers: infrastructure layer, platform layer, and application layer. In addition, there are management and security layers that run through the three layers. The CC architecture is shown in Figure 1.

### 2.4. Digital Sports

#### 2.4.1. Development Status

For the first time in the Fifth Olympic Games, “digital sports” technology was adopted, that is, electronic timing and camera equipment. Currently, digital sports technology has been popularized in sports competitions. For example, the camera during the track and field sprint, the decomposition of figure skaters' movements, the score of basketball, the playback of swimming movements all make full use of the role of BD and CC. Moreover, the playing of online sports is also one of the manifestations of digital sports. The look and feel of VR technology is an exciting experience [9]. The German medilogic company applies the foot-pad type plantar pressure measurement system to sports training and medical rehabilitation. When measuring, it analyzes the athlete's standard of movement and technical movement through the change of the center of gravity, which helps to improve the performance. The American ALTERG space capsule weight-reducing treadmill uses air pressure weight-reduction technology to help athletes lose weight efficiently. In addition to sports powers such as the United States and Germany, some European countries such as Finland and Japan have advanced independent digital sports training equipment. Not only are the technologies mature, but the training methods are also constantly innovating and developing. In recent years, the Chinese government has gradually begun to pay attention to the development of digital sports and has achieved substantial results. It uses computer vision recognition technology or sensor technology to serve groups who desire scientific exercise and healthy diet [10, 11]. Different from the relatively sedentary activity form of simple eyeball + finger in traditional e-sports and online games, digital sports put more emphasis on the “sweating” limb movement. With the help of cameras, wearable helmets or sensors and motion capture systems, interactive sports and entertainment between man and machine and between people, network systems and people can be realized. Almost all traditional sports and entertainment forms can be “decoded” and “coded” again by means of “Digital Sports.” Digital sports iares the upgrading of traditional e-sports. Digital sports are the product of the development of sports, science, and technology.

However, by consulting Chinese academic journals and research literature on physical education teaching in some colleges and universities, it is found that the teaching and training of physical education subjects have the following problems that need to be solved urgently:

1. The teaching method is not scientific. In sports training, physical training is very boring and technical training makes it difficult to master the essentials of movement, which affects many athletes with good physical conditions and affect the training effect due to insufficient comprehension ability. Some sports colleges have realized the importance of reforming educational methods.
2. The selection criteria are not clear. At present, most sports events in our country are based on the selection of professional teams. The basis is a three-level selection system for juvenile teams, youth teams, and national teams, which can ensure the depth and breadth of the selection. The selection of high school students and sports students is based on the sports event. Development is of great significance. In the selection of sports training, removing the influence of human factors, the standard for selection of coaches can only be the performance of the athletes. For example, in track and field, each sport has corresponding results and standards, while football and volleyball are used in the selection of young athletes. At the time, more attention should be paid to the potential of athletes.
3. In professional sports training, sports injuries are the product of unreasonable training methods, training volumes, and wrong training actions. Although it is difficult to completely avoid them, the possibility of injury should be minimized. Although preventing sports injuries is also a compulsory course for professional athletes, the effect of preventing injuries only theoretically is obviously not good. Almost every professional athlete has more or less injuries. Wrong training mode can cause athletes to be injured, and at the worst, it can directly ruin the sports career, especially in the field of selection of young athletes. The large number of athletes and imperfect skills have buried many potential sports talents [12, 13].
4. There is lack of digital sports resources: at present, sports training and teaching are not closely integrated with modern teaching technology, and there are not enough digital sports resources that can be used for training and teaching or as selection criteria. If a quantitative training parameter standard can be formulated, it can provide a reference for the training and selection of athletes, prevent human factors in the coach selection process, create a good environment for the selection of athletes, and avoid burying any sports talent.

#### 2.4.2. Overall Plan for Digital Sports Training

This subject proposes a sports training system; the purpose is to provide solutions for sports workers through posture data, and the system is mainly composed of three parts, namely posture data acquisition module, wireless communication module, and application software.

The first part is the posture data collection node, which is used to capture the posture data of the human body. It is the basis of system analysis and application. The accuracy of the data should be ensured; otherwise, the measurement effect and analysis for athletes or sports events will be meaningless. In the second part, wireless communication module, because the acquisition module is bound to the athlete's body, the number of nodes and the acquisition frequency require that the communication module must ensure that a large AOD can be transmitted and that it is within a certain working range. Part three is the client application software. It would be used to display the athlete's model and three-dimensional scene and also include data display, storage, analysis, and other functions, to provide a friendly interactive interface for coaches or athletes. The fourth part, cloud server, can ensure data security and provide client data with the access of the service.

1. Construction of a human joint model [14]: the construction of a human body model can be used to extract human body posture features and human motion capture, but the basic human body model cannot provide a reference for professional sports training. It should be determined whether the technical movement standard of sports is related to the following aspects: the strength of the tendons, the elasticity of the ligaments, and the range of joint motion. Multiple MPU9250 inertial navigation sensors are used to wear on a certain joint of the athlete's limbs, the posture of the movement is parameterized by the angle and force, and the data of each training process is recorded.
2. Standardization of technical actions: in many sports, skill is more important than strength. Analyze the direction of force transmission. Only when all tendons produce force in the same direction can you achieve better results. It can analyze and compare the data in the movement process, judge the difference between the movement of the limbs and joints and the standard movement, and determine the cause of the wrong movement [15, 16].
3. Early warning of joint damage: there are three main types of motions of human joints, namely flexion and extension, pronation/supination, and circular rotation. Due to the limitations of joint bones, ligaments, and tendons, each type of motion is limited in a specific direction, exceeding the limit position range. Ligaments are easy to strain, and repeated exertion of tendons can also cause fatigue [17]. Combining the content of human physiology can describe the extreme positions of vulnerable joints, and during the monitoring training process, it can remind athletes to reduce joint damage.
4. Fatigue analysis: the wearable sensor detects the human body motion process, and the process parameters can be extracted from it after multiple monitoring. For example, by continuously monitoring the action process of multiple long jumps, analyzing and comparing with the historical data of the athlete's training, and focusing on the analysis of the changing trend of the athlete's action parameters during the consecutive multiple long jumps, it can be judged that the athlete has reached the best after the first few warm-ups state, where it is easy to get good results and reach fatigue state in the first few jumps [18].

### 2.5. Design of the Sports Training Data Monitoring Device

#### 2.5.1. Nonwearable

Nonwearable posture monitoring technology generally refers to a monitoring method in which the monitoring device or system is fixed or noncontact with the human body. During the monitoring process, the human body and the monitoring device will move relative to each other, and the device needs to be powered by an external power supply. Nonwearable monitoring technologies mainly include the following.

1. Optical image recognition technology: at present, the research of human body posture based on optical image monitoring methods is very common, and the technology is relatively mature. The motion posture of the measured object is captured by a camera, the image is taken by an optical monitoring system, and the captured image is analyzed to calculate the posture and motion parameters of the measured object. This monitoring method requires several cameras, including ordinary lenses, infrared cameras, and depth cameras, to be arranged in a specific monitoring site. The essence of this method is pattern recognition. The computer monitors the motion posture of the measured object by tracking and classifying video image sequences. Optical image recognition technology has no effect on the measured object, but the layout scene and equipment requirements are higher. Recognition is mainly based on human facial image features. How to recognize the changes caused by posture has become one of the difficulties of this technology. The pose problem involves the face change caused by the rotation of the head around three axes in the three-dimensional vertical coordinate system, in which the depth rotation in two directions perpendicular to the image plane will cause the partial loss of face information. The attitude problem has become a technical problem.
2. Electromagnetic positioning and tracking technology: the method of human body posture based on electromagnetic wave positioning is also widely used. The monitoring system is composed of a transmitter, a receiver, and a processor. The measurement principle is such that the transmitter emits electromagnetic waves of a certain frequency and the receiver receives the electromagnetic waves. The subject should wear a receiving sensor on a part of the body to monitor the changes in the magnetic induction intensity, according to the coupling relationship between the transmission and reception of electromagnetic induction signals. Analyze the human body movement posture. The electromagnetic positioning and tracking technology does not have much influence on the motion posture of the measured object, but the tracking device is susceptible to electromagnetic interference from other communication equipment.
3. Acoustic positioning and tracking technology: the acoustic-based positioning and tracking method is similar in principle to the electromagnetic positioning and tracking method, except that the measured electromagnetic wave is replaced with the measured acoustic wave. The acoustic monitoring system consists of a sound source, a sound wave receiver, and a processing unit. The principle of acoustic wave measurement is such that multiple acoustic pulses are sent by a sound source, and echoes are generated when the pulse signals reach the object to be measured. And then the acoustic wave receiver receives multiple echo signals, and the object is to be location tracked according to the time difference or phase difference of the reflection. This measurement method has no effect on the movement posture of the measured object, but because the speed of sound waves propagating in the air is relatively low, the real-time performance is poor.

#### 2.5.2. Wearable

Wearable posture monitoring technology means that the posture sensor is worn on the measured object, and the posture of the measured object is determined according to the posture of the sensor. This kind of monitoring technology needs to avoid the influence of wearable sensors on the natural movement of the human body, and it needs autonomous power supply and wireless communication technology. Wearable posture monitoring methods are as follows:

1. Mechanical tracking method: the basic principle of the mechanical tracking method is to determine the relative motion relationship between human body parts according to the relationship between the mechanical structure measurement datum and the measured point. Mechanical structure measurement includes a combination of various sensor parameters such as temperature, acceleration, bending stress, and pressure. The advantages of this measurement method are good real-time performance and strong anti-interference ability, but the shortcomings are also very obvious. The measured object has a greater influence on the movement posture after wearing the mechanical device and loses the authenticity of the monitoring posture, so it is only suitable for static measurement which is difficult to be widely used.
2. Based on sensor monitoring method: with the continuous development of MEMS technology, many types of sensors can be used to measure different parameters. As a revolutionary new technology, with its small size and light weight, it has been widely used in high-tech industries. Using a contact measurement method, the MEMS inertial navigation sensor moves with a specific part of the human body, and each sensor node measures its own motion parameters. There are many kinds of sensors for measuring the posture of the human body, including accelerometers, gyroscopes, and geomagnetometers. It can also be used in a single accelerometer or a combination of multiple sensors to improve the reliability and accuracy of posture detection. The acceleration of the human body parts measured by the inertial sensor node is combined with angular acceleration and geomagnetic parameter compensation to calculate the motion acceleration and azimuth. At present, there are countless products using MEMS inertial navigation sensor technology in the market, and there are more and more users in daily life. Most of them are used for people's fitness. It also reflects the mature development and application prospect of this technology, and the hardware device is convenient to wear and low in cost. MEMS is interdisciplinary. MEMS involves many disciplines such as electronics, machinery, materials, manufacturing, information and automatic control, physics, chemistry, and biology and integrates many cutting-edge achievements in the development of science and technology.

## 3. Research and Development of Virtual Swimming Training Simulation Teaching Device

### 3.1. Overall Demand Analysis

According to the needs of the questions, this paper selected 50 students who took the elective swimming course to conduct a questionnaire survey. The content of the questionnaire includes common problems in swimming training, expectations of swimming lessons, and views on virtual teaching. After sorting out the data, we get Table 2.

As shown in Table 2, of the four basic common problems, insufficient preparation before swimming is the easiest thing to happen. With the end of swimming, 25% of people also said that their ears are prone to water and itching. These problems in swimming classes bring uncomfortable experience to people, so the design of teaching devices for swimming training needs to meet corresponding needs.

By analyzing the problems faced by students in swimming training, and investigating the research status of virtual reality swimming programs and head position tracking technology at home and abroad, in order to ensure the immersion, interaction, and imagination of the virtual swimming training simulation device, the overall design requirements are summarized as follows:

1. Design a suitable support structure to allow the user to float in mid-air in a prone posture to simulate swimming and to provide a basic simulation of buoyancy in the water. Reasonable selection of materials to ensure the safety and comfort of virtual swimming.
2. Determine a reasonable head position detection plan and use the positioning ball group, camera, and computer to complete the automatic detection of the user's head position to ensure the accuracy and real-time performance of the head position detection. Design a suitable positioning ball set to meet the requirements of pose detection while ensuring user comfort.
3. Choose a suitable virtual environment to build software and build a virtual swimming scene to meet the user's freely definable requirements for swimming scenes. Deploy the virtual scene program to the VR headset, reasonably update the field of view according to the received pose data, and visually provide a real virtual swimming experience.

### 3.2. Overall Plan

The overall design block diagram of the virtual swimming training simulation device designed in this subject is shown in Figure 2. The device is composed of a supporting structure, a posture detection system, and a virtual environment system. Among them, the supporting structure is composed of a swimming frame and a suspension device, which is responsible for carrying users and providing simulation of swimming posture and buoyancy in the water. The pose detection system consists of a positioning ball group, a camera, and a head position detection program and is responsible for the automatic detection and data transmission of the user's head position. The virtual environment system is composed of a VR headset and a virtual scene program and is responsible for the presentation of virtual swimming scenes, the reception of head posture data, and the update of the field of view.

### 3.3. Pose Detection Method

In the virtual swimming training simulation device, accurate and real-time detection of the position and posture of the positioning ball group can make the virtual swimming scene change in accordance with the user's movement and head rotation, which is a key step in realizing natural human-computer interaction.

The position and posture of an object in three-dimensional space can be represented by the rotation and translation matrix of its own coordinate system relative to a fixed coordinate system:

(1) $$\begin{array}{c} \left[\begin{array}{c} a_{x}\\ b_{x}\\ c_{x} \end{array}\right]=\left[\begin{array}{c} w_{11},w_{12},w_{13}\\ w_{21},w_{22},w_{23}\\ w_{31},w_{32},w_{33} \end{array}\right]\left[\begin{array}{c} a_{q}\\ b_{q}\\ c_{q} \end{array}\right]+\left[\begin{array}{c} g_{1}\\ g_{2}\\ g_{3} \end{array}\right]=P\left[\begin{array}{c} a_{q}\\ b_{q}\\ c_{q} \end{array}\right]+g. \end{array}$$

In addition to using a rotation matrix, it can also be represented by a quaternion. A quaternion is composed of four elements, which can be seen as a vector in a four-dimensional space or as a hypercomplex number. Its plural expression is as the following formula:

(2) $$\begin{array}{c} P=\left(p_{1},p_{2,}p_{3},p_{4}\right)=p_{1}\overset{⟶}{j}+p_{2}\overset{⟶}{j}+p_{3}\overset{⟶}{j}+p_{4}. \end{array}$$

## 4. Experimental Data Analysis

### 4.1. Classifier Performance Comparison Experiment

In order to achieve the best positioning ball group image recognition effect, this paper conducts positioning ball group classifier training based on LBP, Haar, and HOG features, carries out classifier performance comparison experiments, and selects the best classifier that meets the positioning ball group recognition requirements. The experiment uses two test videos to test the performance of the three classifiers in recognizing the positioning ball group. These two test videos are taken when the user is performing an actual virtual swimming exercise on the virtual swimming training simulator. The total number of frames of video 1 is 1080 frames, the total number of frames of video 2 is 1067 frames, and each frame contains a complete set of positioning ball images. The performance evaluation indicators adopted in the experiment include accuracy rate, recall rate, and target recognition speed (Table 3).

As shown in Figure 3, the classifier using HOG features achieved the highest classification accuracy and recall in the two test videos. In addition, in the subsequent calculation of the coordinates of the feature point image, the negative samples that are incorrectly classified as positive cannot detect four small ball images in the range of different tonal values, which are invalid images, but still require a certain amount of processing time. This has a greater impact on the real-time performance of pose detection. However, the number of invalid images (FP) detected by the classifier using HOG features during performance experiments and actual use is extremely small, which greatly reduces the time required for the overall head position detection process.

### 4.2. Investigation on the Reasons Why People Choose Sports

This article also uses Internet data to analyze the reasons why people choose basketball, badminton, table tennis, and swimming. A total of 256 pieces of data were investigated, and the results are as follows.

As shown in Figure 4, people choose to play basketball, swimming, and table tennis mainly because of interest and entertainment, while the reason for playing badminton is health. These data show that people will consider their effects on people when they choose sports. We can infer that sports activities as a part of people's daily life have its value. Therefore, training in sports should also be indispensable. Therefore, the design and application of physical training teaching devices are undoubtedly an important part of the development of sports in our country.

## 5. Conclusion

At present, the domestic sports training teaching methods are not scientific enough, the selection criteria are not clear, the sports injury is serious, and the digital resources are scarce. Therefore, this article has studied the sports training data monitoring device and design the virtual swimming training simulation teaching device taking swimming as an example. The results show that the use of BD analysis technology to integrate them can better improve the effect of sports training and promote the improvement of the construction of high-quality talents in our country in the future. The requirements of the digital sports training system are basically completed, which can provide solutions for sports training, reduce sports injuries, standardize athletes' movements, and help improve training performance. Moreover, with the development of people's living standards, sports education is becoming more and more important. With the progress of cloud technology, big data analysis becomes more perfect, which brings better results. Cloud helps to integrate data from many sources. It can not only improve analysis, simplify infrastructure, reduce costs, and greatly improve security and privacy.

## Figures and Tables

**Figure 1:** Cloud computing architecture platform.

**Figure 2:** Overall design of the swimming training device.

**Figure 3:** Comparison of accuracy and recall in classifiers.

**Figure 4:** Reasons for choosing different sports items.

**Table 1:** Sports item.

Numbering	Items
01	Swim
02	Archery
03	Track and field
04	Badminton
05	Basketball
06	Boxing
07	Bicycle
08	Gymnastics
09	Volleyball
10	Ping-pong
11	Weightlifting
12	Wrestling
13	Football
14	Tennis
15	Triathlon
16	Fence
...	...

**Table 2:** Common problems in swimming and overall requirements for virtual teaching devices.

	Insufficient preparation (%)	Stay too long (%)	Eyes itching (%)	Water enter into ears (%)
Supporting structure	28	21	27	25
Head pose detection	24	33	26	17
Virtual environment building software	18	30	24	28

**Table 3:** Classifier performance comparison experiment results.

Video sequence number	Feature type	Tp	FP	Accuracy (%)	Recall rate (%)	Operation hours (s)
1	LBP	832	134	83.56	78.25	40.18
	Haar	857	128	86.37	84.21	46.58
	HOG	896	33	95.89	87.66	53.12

2	LBP	786	264	74.39	73.62	37.85
	Haar	839	145	86.14	80.09	44.32
	HOG	917	39	94.59	84.67	50.69

## Data Availability

The data underlying the results presented in the study are included within the manuscript.
